The article "San-Huang-Chai-Zhu Formula Ameliorates Liver Injury in Intrahepatic Cholestasis through Suppressing SIRT1/PGC-1α-Regulated Mitochondrial Oxidative Stress" was published in 2022. Journal: Evid Based Complement Alternat Med.

# San-Huang-Chai-Zhu Formula Ameliorates Liver Injury in Intrahepatic Cholestasis through Suppressing SIRT1/PGC-1*α*-Regulated Mitochondrial Oxidative Stress

**DOI:** 10.1155/2022/7832540

**Published:** 2022-07-08

**Authors:** Binbin Liu, Jie Zhang, Lu Shao, Jiaming Yao

**Affiliations:** Department of Digestion, Hangzhou TCM Hospital Affiliated to Zhejiang Chinese Medical University, Hangzhou 310007, China

## Abstract

**Background:**

Chinese herbal formulae possess promising applications in treating intrahepatic cholestasis.

**Objective:**

Our study aims to explore the protective effect of the San-Huang-Chai-Zhu formula (SHCZF) on liver injury in intrahepatic cholestasis (IC) and investigate the underlying mechanism related to mitochondrial oxidative stress.

**Methods:**

An IC rat model was established by *α*-naphthyl isothiocyanate induction. Hepatic histomorphology was observed through hematoxylin and eosin staining. Levels of biochemical indexes of hepatic function and oxidative stress were determined by an enzyme-linked immunosorbent assay. Cell apoptosis in liver tissues was detected by the TUNEL assay. The mRNA expression of mtDNA, SIRT1, and PGC-1*α* was measured by qRT-PCR, and the protein expression of Bax, Bcl-2, caspase-3, SIRT1, and PGC-1*α* was determined by Western blotting.

**Results:**

SHCZF treatment attenuated liver injury in IC. Levels of hepatic function parameters were decreased after SHCZF administration. In addition, the decreased level of malondialdehyde (MDA) and the increased levels of superoxide dismutase (SOD), glutathione (GSH), and adenosine triphosphate (ATP) in hepatic mitochondria confirmed that SHCZF could attenuate oxidative stress in IC. SHCZF treatment also reduced the apoptosis in the liver tissues of IC rats. Furthermore, SHCZF administration upregulated the expression of mtDNA, SIRT1, and PGC-1*α* in IC.

**Conclusions:**

SHCZF exerts a protective effect on liver injury in IC via alleviating SIRT1/PGC-1*α*-regulated mitochondrial oxidative stress.

## 1. Introduction

Intrahepatic cholestasis (IC) is a common clinical disease of the digestive system, which is mainly triggered by hepatocyte dysfunction or bile duct obstruction [1, 2]. IC is mostly found in pregnant women, accounting for 0.2–2% of all complications in pregnancies [3]. Long-term IC will progress to liver fibrosis and even cirrhosis, leading to a series of liver diseases such as primary biliary cirrhosis, primary sclerosing cholangitis, and biliary atresia [4, 5]. At present, some drugs, such as rosiglitazone, obeticholic acid, and ursodeoxycholic acid (UDCA), are commonly used for IC treatment. However, they may contribute to dyslipidemia and gastrointestinal symptoms [6–8]. Therefore, the discovery of new drugs for IC treatment is urgently needed.

Recently, Chinese herbal formulae have been increasingly used in the treatment of IC and have exerted a dramatic effect [9–11]. The San-Huang-Chai-Zhu formula (SHCZF), a traditional Chinese herbal formula, consists of Dahuang (*Rhei Radix et Rhizoma*), Huangbai (*Phellodendri Chinensis Cortex*), Huangzhizi (*Gardeniae Fructus*), Chaihu (*Bupleuri Radix*), and Baizhu (*Atractylodis Macrocephalae Rhizome*) [12]. These 5 herbs in SHCZF all exerted a hepatoprotective effect on liver diseases. Among them, emodin (an anthraquinone compound) from Dahuang exerts a critical hepatoprotective effect on IC via antioxidation and promotes bile acid secretion [13, 14]. Demethyleneberberine from Huangbai can effectively ameliorate mitochondrial dysfunction and oxidative stress in alcoholic liver disease [15]. Through the network pharmacology analysis, iridoid glycosides from Huangzhizi play a critical pharmacological role in liver diseases by regulating inflammation [16]. Chaihu as a meridian-inducing medicine is generally utilized in the treatment of liver diseases when combined with other Chinese herbal medicines [17]. Baizhu also has a protective effect on liver injury and oxidative stress [18, 19]. In addition, our previous study has confirmed that SHCZF obviously relieved liver injury in IC rats [12]. However, the underlying mechanism by which SHCZF alleviates IC has not been fully elucidated.

Oxidative stress is a common feature in most hepatopathies [20, 21]. The excessive production of reactive oxygen species (ROS) stimulated by oxidative stress decreases antioxidative capacity and induces hepatic stellate cell proliferation, thereby resulting in liver injury in liver diseases, including IC [22, 23]. Mitochondria are the major sites of oxidative metabolism and the main energy source in hepatocytes, involved in maintaining liver function [24]. ROS overproduction in hepatic mitochondria can destroy the balance of oxidation and antioxidation and contribute to mitochondrial dysfunction and oxidative stress in IC. Some evidence supports that some specific drugs, such as magnesium sulphate and dioscin, exert a therapeutic effect on IC through alleviating mitochondrial dysfunction and oxidative stress [25, 26]. Additionally, peroxisome proliferator-activated receptor gamma coactivator-1*α* (PGC-1*α*) activated by deacetylase sirtuin1 (SIRT1) is a critical regulator of mitochondrial biogenesis and function and oxidative stress [27–29]. Massive existing evidence indicates that liver injury can be attenuated by activating the SIRT1/PGC-1*α* pathway to promote mitochondrial biogenesis and alleviate oxidative stress in liver diseases [30–32]. However, it remains unclear whether SHCZF mitigates oxidative stress via regulating the SIRT1/PGC-1*α* signaling pathway, thereby treating IC.

In this article, we studied the therapeutic effect of SHCZF on IC by evaluating hepatic function and oxidative stress. Meantime, the underlying mechanism of SHCZF regulating the SIRT1/PGC-1*α* pathway was uncovered. These findings reveal the underlying mechanism of SHCZF against IC and provide a new drug to treat IC.

## 2. Materials and Methods

### 2.1. Experimental Animals

Animal experiments were approved by the Animal Experiment Ethics Committee of Hangzhou TCM Hospital Affiliated to Zhejiang Chinese Medical University. Male Sprague Dawley rats (*n* = 48, aged 8 weeks, 200 ± 20 g; Chengdu Dossy Experimental Animals CO., LTD., China) were adaptively raised in an experimental animal room with a 12 h light/dark cycle at 22°C. After one week, rats were randomly divided into 6 groups (*n* = 8): the normal group; the model group; the low-dose SHCZF group; the mid-dose SHCZF group; the high-dose SHCZF group; and the positive control group. Rats in the normal group were gavaged with 0.5% sodium carboxymethyl cellulose. Rats in low-, mid-, high-dose SHCZF, and positive control groups were respectively given 2.5 g/kg, 5 g/kg, 10 g/kg SHCZF, and 90 mg/kg UDCA by gavage. Five days later, rats in the model, low-, mid-, high-dose SHCZF, and positive control groups were gavaged with 100 mg/kg *α*-naphthyl isothiocyanate (ANIT) dissolved in sesame oil to induce IC in rats. After treatment, all rats were anesthetized via intraperitoneal injection with 50 mg/kg pentobarbital sodium and then sacrificed by cervical dislocation. Hepatic tissues and serum samples were collected.

### 2.2. Hematoxylin and Eosin (H&E) Staining

H&E staining was performed as previously described [33]. Briefly, hepatic tissues were fixed with 10% formaldehyde for 48 h and dehydrated with alcohol. Then, tissues were embedded in paraffin and cut into 4 *μ*m-thick sections using the Leica RM2235 rotary microtome (Leica, Germany). After being deparaffinized and rehydrated with alcohol, sections were stained with hematoxylin for 5 min, followed by eosin for 1-2 min. Hepatic tissue sections were subsequently observed and imaged under a light microscope (Olympus, Japan).

### 2.3. Determination of Hepatic Functions

Removed hepatic tissues and serum were utilized for the assessment of hepatic function by an enzyme-linked immunosorbent assay (ELISA). Levels of hepatic function parameters, including alanine aminotransferase (ALT), aspartate aminotransferase (AST), *γ*-glutamyl transpeptidase (GGT), lactate dehydrogenase (LDH), and alkaline phosphatase (ALP), were measured using corresponding ELISA kits (Elabscience, China) in accordance with the manufacturer's instructions. In addition, the contents of IC indexes, including total bilirubin (TBiL) and total bile acid (TBA), were determined using corresponding ELISA kits (Elabscience).

### 2.4. Fractionation and Identification of Hepatic Mitochondria

Mitochondrial fractionation was conducted for the functional identification of hepatic mitochondria. Briefly, hepatic tissues were incubated in isolation buffer (2 mmol/L HEPES, 0.5 mmol/L EGTA, 70 mmol/L mannitol, 220 mmol/L sucrose, and 0.1% bovine serum albumin, pH 7.4; tissue: buffer (w*/*v) = 10 : 1). After homogenate, unbroken cells and nuclei were precipitated by centrifugation at 1,000 × *g*, 4°C for 10 min. The supernatant was centrifuged at 10,000 × *g*, 4°C for 10 min, and pellets were collected as mitochondrial fractions. For assessment of mitochondrial function and oxidative stress, the contents of malondialdehyde (MDA), superoxide dismutase (SOD), glutathione (GSH), adenosine triphosphate (ATP), and 8-hydroxy-2-deoxyguanosine (8-OHdG) were determined using corresponding ELISA kits (Elabscience).

### 2.5. TUNEL Apoptosis Analysis

Liver tissues of rats were subjected to a TUNEL assay to determine apoptosis. Briefly, liver tissues were fixed in 10% formalin and then embedded in paraffin. Next, embedded tissues were sectioned at a 5 *μ*m thickness, followed by dewaxing in xylene for 10 min and rehydrating in gradient ethanol. After washing with phosphate buffered saline (PBS) trice, sections were stained with the reagent from the One Step TUNEL Apoptosis Assay Kit (Beyotime, China) for 1 h at 37°C in darkness. The cytoplasm was stained with 10 *μ*g/mL of 4′, 6-diamidino-2-phenylindole (DAPI). Finally, the apoptosis of liver tissues was observed using a fluorescence microscope (Shanghai optical instrument factory, China).

### 2.6. Quantitative Real-Time (qRT)-PCR

Total RNA was extracted from hepatic tissues using Trizol reagent (Invitrogen, CA, USA), and cDNA was synthesized via reverse transcription using First-Strand cDNA Synthesis SuperMix (TransGen, China). qRT-PCR was performed using the SYBR® Premix Ex Taq™ II (TaKaRa, Japan) in the Mx3000P Real-Time PCR System (Stratagene, CA, USA). The reaction program was as follows: 95°C for 3 min, and 40 cycles of 95°C for 12 s, and 62°C for 40 s. Primers are listed in Table 1. The expression of genes was calculated using the 2^−∆∆Ct^ method and normalized to GAPDH.

### 2.7. Western Blot

Total protein was extracted from hepatic tissues using radioimmunoprecipitation (RIPA) lysis buffer containing a phenylmethanesulfonylfluoride (PMSF) protease inhibitor mixture (Sigma-Aldrich, MD, USA) at 4°C for 15 min. A BCA Protein Assay Kit (Thermo Fisher Scientific, CA, USA) was used to determine the protein concentration. Proteins were separated by 10% SDS-PAGE and then transferred onto polyvinylidene difluoride membranes for 2 h at 65 V. Membranes loaded with target proteins were incubated with blocking buffer (5% skim milk dissolved in 1× Tris buffered saline with 0.1% tween-20 (1× TBST)) for 1 h and then incubated with primary antibodies Bax (1 : 1,000; No. ab32503, Abcam, UK), Bcl-2 (1 : 500; No. ab196495, Abcam), caspase-3 (1 : 2,000; No. ab184787, Abcam), SIRT1 (1 : 1,000; No. ab189494, Abcam), PGC-1*α* (1 : 500; No. AF5395, Affinity Biosciences, OH, USA), and GAPDH (1 : 10,000; No. ab181603, Abcam) at 4°C overnight. Followed by that, membranes were incubated with secondary antibody goat anti-rabbit IgG H&L (HRP) (1 : 2,000; No. ab205718, Abcam) for 1 h in the dark. Protein bands were presented by the ECL reagent kit (Thermo Fisher Scientific) and photographed with a ChemiDoc™ imaging system (Bio-Rad, CA, USA). Relative protein expression was quantified by calculating the band density normalized to GAPDH.

### 2.8. Immunohistochemistry

Hepatic tissues were embedded in paraffin and sectioned at a 4-*μ*m thickness for immunohistochemical staining. Before staining, antigen retrieval was conducted using a citric acid buffer at 126°C for 2 min in a pressure cooker. Then, hepatic tissues were blocked in 3% H_2_O_2_ for 20 min to restrain endogenous peroxidase activity, followed by incubation with normal goat serum for 15 min. Next, sections were incubated with antirabbit SIRT1 primary antibody (1 : 500, Abcam) for 30 min at 4°C and then with anti-goat HRP-labeled secondary antibody (1 : 50, MultiSciences) for 15 min. After incubation with streptavidin peroxidase for 15 min, sections were stained with diaminobenzidine (DAB) using a DAB substrate kit (Changdao, China) and counterstained with hematoxylin (BASO, China) for 3 min. Subsequently, sections were dehydrated, mounted with neutral resin, and observed under a light microscope (Olympus, Japan).

### 2.9. Statistical Analysis

Each experiment was conducted in triplicate. All data were expressed as the mean ± standard deviation. Statistical analysis was performed on SPSS 27.0 (IBM, NY, USA). Intergroup comparisons were carried out using a one-way analysis of variance (ANOVA), followed by Tukey's test. *P* < 0.05 was considered as the indicator of a statistically significant difference.

## 3. Results

### 3.1. SHCZF Alleviated Hepatic Injury in IC

An IC rat model was established by gavage with ANIT (a hepatotoxic agent). H&E staining revealed intracytoplasmic bile pigment deposition, inflammatory cell infiltration, and bile duct dilatation in the hepatic tissues of IC rats compared with normal rats (Figures 1(a) and 1(b)). After SHCZF administration, these histopathological features markedly ameliorated in a dose-dependent manner (Figures 1(c)–1(e)). UDCA is a hydrophilic biliary acid widely used to treat IC. Here, results showed that the mid- and high-dose SHCZF presented a similar hepatoprotective effect with UDCA (Figures 1(d)–1(f)).

### 3.2. SHCZF Protected the Hepatic Function in IC

Serum levels of hepatic injury markers, including ALT, AST, GGT, LDH, and ALP, were measured to assess the hepatoprotective effect of SHCZF. Compared with those in normal rats, the levels of these markers were significantly increased in IC rats (*P* < 0.01) (Figures 2(a)–2(e)). SHCZF treatment effectively reduced the levels of these hepatic biochemical indicators in a dose-dependent manner (*P* < 0.05). Moreover, treatment of high-dose SHCZF showed a more excellent protective effect on liver injury in IC rats than in the positive control group (*P* < 0.05). TBiL and TBA, the main serum indexes for IC, were also determined to evaluate the therapeutic effect of SHCZF. The levels of TBiL and TBA were dramatically increased in IC rats compared with those in normal rats (*P* < 0.01) (Figures 2(f) and 2(g)). SHCZF administration dose-dependently decreased the levels of TBiL and TBA in IC rats (*P* < 0.05). In addition, compared with the positive control, high-dose SHCZF evidently exhibited a better therapeutic effect on IC (*P* < 0.05).

Mitochondrial dysfunction and oxidative stress are associated with the pathogenesis of IC. Levels of oxidative stress indicators, including MDA, SOD, GSH, and ATP, were determined to evaluate the oxidative damage in IC. The content of MDA in IC rats was significantly increased compared with that in normal rats (*P* < 0.001), whereas SHCZF treatment concentration-dependently decreased the level of MDA in IC rats (*P* < 0.05) (Figure 3(a)). The high-dose SHCZF administration showed a better effect than UDCA (*P* < 0.01). In addition, a significant reduction of antioxidants, including SOD, GSH, and ATP, was observed in IC rats compared with that in normal rats (*P* < 0.01) (Figures 3(b)–3(d)). SHCZF treatment markedly increased the levels of SOD, GSH, and ATP in IC rats in a dose-dependent manner (*P* < 0.05). The antioxidative effect of high-dose SHCZF was superior to UDCA (*P* < 0.05). 8-OHdG, a DNA oxidative damage marker, was dramatically increased in the hepatic mitochondria of IC rats compared with that in normal rats (*P* < 0.01). Similarly, SHCZF treatment dose-dependently reduced the level of 8-OHdG in IC rats (*P* < 0.05) (Figure 3(e)). Furthermore, mtDNA is highly sensitive to mitochondrial dysfunction and oxidative stress. Compared with that in normal rats, the expression level of mtDNA in hepatic tissues of IC rats presented a significant decrease (*P* < 0.01). SHCZF administration obviously promoted the expression of mtDNA in IC rats in a dose-dependent manner (*P* < 0.05). High-dose SHCZF and UDCA treatment presented a similar effect on upregulating the expression of mtDNA (Figure 3(f)).

We further investigated the effects of SHCZF on apoptosis in the hepatic tissues of IC rats. The TUNEL assay showed that the cell apoptosis in the liver tissues of IC rats obviously increased when compared with that in normal rats. After SHCZF or UDCA treatment, cell apoptosis in liver tissues of IC rats was reduced in a dose-dependent manner (Figure 4(a)). In addition, the pro-apoptotic protein (Bax) and the antiapoptotic protein (Bcl-2) are the crucial regulators of cell apoptosis [34]. Markedly increased Bax level and decreased Bcl-2 level were observed in the liver tissues of IC rats compared with those in normal rats (*P* < 0.01). The expression of caspase-3 (another apoptosis biomarker) was also shown to be higher in IC rats than in normal rats (*P* < 0.01). However, levels of Bax and caspase-3 were decreased, and Bcl-2 level was increased in IC rats by SCHCZF or UDCA administration (*P* < 0.05) (Figure 4(b)).

### 3.3. SHCZF Activated the SIRT1/PGC-1*α* Pathway in IC

The SIRT1/PGC-1*α* signaling pathway is involved in mitochondrial biogenesis and protection. As shown in Figures 5(a)–5(e), the expression levels of SIRT1 and PGC-1*α* were remarkably downregulated in IC rats compared with that in normal rats (*P* < 0.01). SHCZF treatment significantly upregulated the expression of SIRT1 and PGC-1*α* in IC rats in a dose-dependent manner (*P* < 0.05). In addition, different doses of SHCZF treatment all exhibited a better effect on activating the SIRT1/PGC-1*α* pathway than UDCA (*P* < 0.001). Furthermore, immunohistochemical staining confirmed that SHCZF treatment dose-dependently upregulated the expression of SIRT1 located in hepatocyte nuclei (Figure 6).

## 4. Discussion

Intrahepatic cholestasis (IC) is manifested as the immoderate accumulation of bile acids in the liver, mainly caused by bile secretion disorders, which is the most common liver disorder in pregnant women [8, 35]. Progressive IC has an increased risk of hepatocellular carcinoma [36, 37]. In recent years, Chinese herbal formulae have become increasingly popular worldwide for treating IC due to their favorable efficacy and low risk. In this study, we found that the Chinese herbal formula SHCZF has the efficacy of ameliorating liver injury and oxidative stress in IC. Besides, the underlying mechanism of SHCZF against IC is involved in the activation of the SIRT1/PGC-1*α* signaling pathway.

SHCZF consists of 5 herbal medicines, including Dahuang (*Rhei Radix et Rhizoma*), Huangbai (*Phellodendri Chinensis Cortex*), Huangzhizi (*Gardeniae Fructus*), Chaihu (*Bupleuri Radix*), and Baizhu (*Atractylodis Macrocephalae Rhizome*) [12]. Previous studies showed that numerous active components in these medicines exhibited obvious protective effects on liver diseases, such as emodin, demethyleneberberine, polysaccharides, and so on [13, 17, 18, 38–40]. SHCZF exhibited a mitigative effect on ANIT-induced acute IC in rats [41]. The application of rodent models is important for the therapeutic and translational research of cholestatic liver disease [42]. In this work, an IC rat model was established by ANIT induction to investigate the hepatoprotective effect of SHCZF. Results showed that there was severe liver structure disorder and cholestasis in the hepatic tissues of IC rats, which is in accordance with previous studies [2, 43]. SHCZF treatment effectively attenuated these pathological conditions, indicating that SHCZF has a hepatoprotective effect on liver injury in IC. ALT, AST, GGT, LDH, and ALP are hepatocyte and serum enzymes basically used as indicators for hepatocyte damage and liver diseases [2]. TBiL and TBA are the indirect indexes that confirm hepatocyte damage, cholestasis, and hepatic dysfunction [44]. Here, levels of these hepatic function parameters presented a decreasing trend after SHCZF treatment, suggesting that SHCZF can alleviate liver injury in IC.

Oxidative stress is a key factor accompanied by liver injury in IC [23]. The occurrence of oxidative stress is related to the production of ROS in mitochondria [45]. Excessive ROS in the liver can lead to an imbalance of oxidation and antioxidation and mitochondrial dysfunction, thereby causing liver injury in IC. Meanwhile, oxidative stress can promote lipid peroxidation, thereby resulting in the increase of MDA (a lipid peroxidation byproduct) level and the relative decrease of SOD (an antioxidant enzyme) [46]. The cellular oxidants GSH and ATP are also critical to defending oxidative stress [47]. In this study, we found that SHCZF treatment markedly reduced the level of MDA and increased the contents of SOD, GSH, and ATP in IC rats. This result indicates that SHCZF has a mitigative effect on oxidative stress and mitochondrial dysfunction in IC. In addition, 8-OHdG is a DNA oxidative damage marker, representing the degree of oxidative stress. MtDNA encodes the genetic information in the mitochondrion, the integrity of which must be maintained to protect mitochondrial function [48]. SHCZF treatment reduced the level of 8-OHdG and increased mtDNA expression in IC rats, illustrating that SHCZF can ameliorate mitochondrial oxidative stress, thereby protecting mitochondrial function in IC. Moreover, hepatocyte apoptosis is also an important pathological feature of IC [26]. In our study, SHCZF markedly downregulated the expression of pro-apoptotic biomarkers (Bax and caspase-3) and upregulated the antiapoptotic marker (Bcl-2) level in the liver tissues of IC rats. This result indicates that SHCZF can reduce the apoptosis in the liver tissues of IC.

The SIRT1/PGC-1*α* signaling pathway is an important regulator of hepatic mitochondrial function. PGC-1*α* is a central hub in mitochondrial biogenesis via interacting with downstream factors including peroxisome proliferator-activated receptors, nuclear respiratory factors, and mitochondrial transcription factors. Interactions of PGC-1*α* and downstream factors activate the expression of mitochondrial proteins [49]. SIRT1 is an upstream gene of PGC-1*α* that regulates PGC-1*α* activity via deacetylation and phosphorylation, thereby affecting mitochondrial function [50]. Accumulating evidence indicates that the SIRT1/PGC-1*α* pathway is involved with liver injury via regulating mitochondrial function and oxidative stress [50–52]. In addition, numerous studies of drugs against liver injury focus on the activation of the SIRT1/PGC-1*α* pathway. For instance, nicotinamide riboside exerts protective effects on alcohol-induced liver injury via activating the SIRT1/PGC-1*α*-mitochondrial biosynthesis pathway [30]. The underlying mechanism of salvianolic acid B mitigating sepsis-induced liver injury is associated with the activation of the SIRT1/PGC-1*α* pathway [31]. Betanin ameliorated cisplatin-induced liver injury through modulating the SIRT1/PGC-1*α* pathway [32]. Our study found that SHCZF administration increased the expression of SIRT1 and PGC-1*α* in IC. Therefore, we speculate that SHCZF attenuates oxidative stress and mitochondrial dysfunction via activation of the SIRT1/PGC-1*α* pathway, thereby protecting hepatic function in IC. Our present study provides a promising therapeutic drug (SHCZF) and target (SIRT1/PGC-1*α* pathway) for IC.

## 5. Conclusions

SHCZF is a potential drug to ameliorate liver injury in IC via alleviating mitochondrial oxidative stress that may be regulated by the SIRT1/PGC-1*α* pathway. This research provides a new drug for IC treatment and sheds light on further study to explore the underlying mechanism of SHCZF therapy. However, there are several limitations to our study: (1) the underlying mechanism of SHCZF regulating the SIRT1/PGC-1*α* signaling pathway has not been fully elucidated; (2) the therapeutic effect of SHCZF against IC still needs to be verified in the clinical trial; and (3) it is still elusive whether other regulators are involved in the mechanism of SHCZF against IC.

## Figures and Tables

**Figure 1:** Hepatic histology was identified by hematoxylin and eosin (H&E) staining. (a) The normal group; (b) the model group (100 mg/kg ANIT); (c) the low-dose SHCZF (2.5 g/kg) group; (d) the mid-dose SHCZF (5 g/kg) group; (e) the high-dose SHCZF (10 g/kg) group; (f) the positive control group (60 mg/kg UDCA). Scale bar = 50 *μ*m.

**Figure 2:** Hepatic function was assessed by the ELISA test. (a) Aminotransferase (ALT) level; (b) aspartate aminotransferase (AST) level; (c) *γ*-glutamyl transpeptidase (GGT) level; (d) lactate dehydrogenase (LDH) level; (e) alkaline phosphatase (ALP) level; (f) total bilirubin (TBiL) level; (g) total bile acid (TBA) level. ^*∗*^*P* <  0.05, ^*∗∗*^*P* <  0.01 and ^*∗∗∗*^*P* < 0.001 vs. the normal group. ^#^*P* < 0.05 and ^##^*P* < 0.01 vs. the model group. ^Δ^*P* <  0.05, ^ΔΔ^*P* < 0.01 and ^ΔΔΔ^*P* < 0.001 vs. the high-dose SHCZF group. SHCZF ameliorated mitochondrial dysfunction and oxidative stress in IC.

**Figure 3:** Hepatic mitochondrial function and oxidative stress were assessed by the ELISA test. (a) Malondialdehyde (MDA) level; (b) superoxide dismutase (SOD) level; (c) glutathione (GSH) level; (d) adenosine triphosphate (ATP) level; (e) 8-hydroxy-2′-deoxyguanosine (8-OHdG) level. (f) The relative mRNA expression of mtDNA in hepatic tissues was measured by qRT-PCR. ^*∗*^*P* <  0.05, ^*∗∗*^*P* <  0.01 and ^*∗∗∗*^*P* < 0.001 vs. the normal group. ^#^*P* < 0.05 and ^##^*P* < 0.01 vs. the model group. ^Δ^*P* <  0.05, ^ΔΔ^*P* < 0.01 and ^ΔΔΔ^*P* < 0.001 vs. the high-dose SHCZF group. SHCZF promoted apoptosis in the hepatic tissues of IC rats.

**Figure 4:** SHCZF reduced cell apoptosis in the liver tissues of IC rats. (a) The cell apoptosis in the liver tissues of rats was determined by the TUNEL assay. Scale bar = 50 *μ*m. (b) The protein expression of Bax, Bcl-2, and caspase-3 in the liver tissues of rats was measured by western blotting. ^*∗∗*^*P* < 0.01 and ^*∗∗∗*^*P* < 0.001 vs. the normal group. ^#^*P* < 0.05 and ^##^*P* < 0.01 vs. the model group. ^Δ^*P* < 0.05 and ^ΔΔ^*P* < 0.01 vs. the high-dose SHCZF group.

**Figure 5:** SHCZF activated the SIRT1/PGC-1*α* signaling pathway. (a–e) The relative mRNA and protein expression of SIRT1 and PGC-1*α* in hepatic tissues was measured by qRT-PCR and Western blotting, respectively. ^*∗*^*P* < 0.05 and ^*∗∗*^*P* < 0.01 vs. the normal group. ^#^*P* < 0.05 and ^##^*P* < 0.001 vs. the model group. ^Δ^*P* < 0.05 and ^ΔΔΔ^*P* < 0.001 vs. the high-dose SHCZF group.

**Figure 6:** The expression of SIRT1 in hepatic tissues was observed by immunohistochemistry. (a) The normal group; (b) the model group; (c) the low-dose SHCZF group; (d) the mid-dose SHCZF group; (e) the high-dose SHCZF group; (f) the positive control group. Scale bar = 50 *μ*m.

**Table 1:** Primer sequences for qRT-PCR.

Gene	Forward (5′-3′)	Reverse (5′-3′)
MtDNA	CCCAACACAGGCGTGCTT	ACCGCGGCCGTTTAACTT
SIRT1	GTTGTGTGCCTTCGTTTTGGA	AGGCCGGTTTGGCTTATACA
PGC-1*α*	GCACCAGAAAACAGCTCCAA	TTGCCATCCCGTAGTTCACT
GAPDH	ACCGCGGCCGTTTAACTT	CCTAGCCCCAGGGCTTTGATT

## Data Availability

The data used to support the findings of this study are available from the corresponding author upon request.
